# Perioperative Effect of Single-Port Thoracoscopic Segmentectomy and Three-Port Thoracoscopic Segmentectomy in the Treatment of Early Non-Small-Cell Lung Cancer

**DOI:** 10.1155/2023/7550317

**Published:** 2023-02-23

**Authors:** Cong Zhang, Dexiong Jiang, Cuilian Luo, Dongdong Yuan, Guansheng Shang

**Affiliations:** ^1^Department of Thoracic Surgery, Chengdu Seventh People's Hospital, Chengdu, 610200 Sichuan, China; ^2^Department of Oncology, Chengdu Seventh People's Hospital, Chengdu, 610200 Sichuan, China

## Abstract

**Background:**

Clinically, there were few reports on single-hole thoracoscopic segmental resection in non-small-cell lung cancer (NSCLC), and no report on the comparison of single-hole and three-hole thoracoscopic segmental resection. Hence, the purpose of the study was to explore the perioperative role of single-port thoracoscopic segmentectomy and three-port thoracoscopic segmentectomy for early-stage NSCLC.

**Methods:**

The clinical data of 80 patients with early-stage NSCLC who were treated in our hospital from January 2021 to June 2022 were selected as the retrospective research subjects and divided into a comparison/research group with 40 cases in each group according to different surgical methods. Among them, the comparison group was received three-port thoracoscopic segmentectomy, and the research group was received single-port thoracoscopic segmentectomy. The surgical indicators, immune and tumor marker levels, as well as prognostic complications between two groups were compared.

**Results:**

There was no remarkable diversity between the two groups in terms of operation time and the number of lymph nodes dissected during the operation (*P* > 0.05). The surgical blood loss in research group was lower than comparison group (*P* < 0.05). After treatment, the levels of CYFRA21-1, CA125, as well as VGEF in the research group were markedly lower than comparison group (*P* < 0.05). The differences in CD^4+^, CD^3+^, and CD^4+^/CD^8+^ after treatment were prominent, and the research group was higher than comparison group (*P* < 0.05). There was no statistical difference in postoperative complications between the two groups (*P* > 0.05).

**Conclusions:**

Single-hole thoracoscopic lobectomy has obvious advantages in the treatment of NSCLC, which can reduce intraoperative bleeding, enhance the recovery of patients' immune function, and promote postoperative recovery.

## 1. Introduction

Non-small-cell lung cancer (NSCLC) is a relatively common clinical malignant tumor of the respiratory system. The incidence rate accounts for about 80% of all lung cancer patients. The mortality rate of patients after diagnosis is high, and it increases year by year with the passage of time [1]. Surgery, as a common method for the treatment of NSCLC, has gradually transitioned from traditional thoracoscopic lobectomy to segmentectomy after years of technological development [2]. At present, three-port thoracoscopy was commonly used in clinical treatment of patients with NSCLC, but there were still shortcomings such as obvious postoperative pain and thoracic movement disorders [3]. In recent years, single-port thoracoscopic segmentectomy, which was characterized by smaller chest wall incisions and more preservation of lung tissue, had been selectively applied in the surgical treatment of patients with NSCLC, especially for peripheral stage I lung cancer. It has been proved that its short-term clinical efficacy was basically the same as that of the three-hole method [3]. However, there were few reports on the single-hole method at present and comparative studies between single hole and three hole.

In the field of segmentectomy for early-stage NSCLC, the more traditional surgical method is the three-port method, including the observation port, the main operating port, and the auxiliary operating port [4, 5]. Although this traditional surgical method had become more and more mature, but massive scholars have found that there were some defects in three-port thoracoscopic surgery, such as numbness or dyskinesia at the distal end of the chest wall, and pain in the auxiliary operating port of the back [6, 7]. So, the single-port thoracoscopic technique came into being, and it was also a major breakthrough in the minimally invasive technique of thoracic surgery in recent years [8]. Single-port thoracoscopic surgery usually chose the fourth or fifth intercostal space between the anterior axillary line and the midaxillary line as the only surgical incision, which was more suitable for the operation angle during the operation. The characteristic of single-port thoracoscope was that various surgical instruments and endoscopic lenses needed to be placed in the same incision, and the operating angle of view was closer to that of open surgery under direct vision, so the relative visual error was small [9].

Hence, the study aimed to seek the perioperative role of single-port thoracoscopic segmentectomy and three-port thoracoscopic segmentectomy for early-stage NSCLC, supplying a fresh direction for clinical treatment of NSCLC.

## 2. Material and Methods

### 2.1. Research Object

The clinical data of 80 patients with early-stage NSCLC who were treated in our hospital from January 2021 to June 2022 were selected as the retrospective research subjects and divided into a comparison/research group with 40 cases in each group according to different surgical methods. Diagnostic criteria were referred to Chinese Medical Association Lung Cancer Clinical Diagnosis and Treatment Guidelines [10].

### 2.2. Inclusion and Exclusion Criteria

Inclusion criteria are as follows: (1) chest high resolution CT (HRCT) showed that the tumor diameter was 2 cm or less, the solid component was less than 50%, and the intraoperative rapid freezing and postoperative pathological diagnosis were NSCLC; (2) cranio-thoracic T, radioactive radionuclide whole-body bone scintigraphy, abdominal color Doppler ultrasound, and other related examinations confirm that the tumor had no distant metastasis; (3) the tumors were all single lesions, and the resection margins of lung tissue were more than 2 cm away from the lesion edge; (4) The general condition of the patient was good, and the patient could tolerate segmentectomy under general anesthesia.

Exclusion criteria are as follows: (1) history of thoracic trauma, or a history of preoperative radiotherapy and chemotherapy; (2) combined with other malignant tumors; (3) central lung cancer or peripheral lung cancer with multiple lesions; (4) patients with underlying diseases such as severe diabetes and hypertension.

### 2.3. Surgical Methods

After admission, the patients in the two groups were inquired about the medical history in detail, carried out a general physical examination, assessed the patient's condition and general physical condition, and improved the relevant preoperative examinations. Preoperative related examinations included blood routine, liver and kidney function, blood type identification, blood coagulation routine, and electrolyte routine as well as routine before blood transfusion. Auxiliary examinations included head CT, chest CT, abdominal ultrasound, cardiac ultrasound, pulmonary function, electrocardiogram, and radionuclide system bone imaging. After the contraindications for surgery were excluded, the surgical treatment was performed. The patients' family members were interviewed before surgery, and the patients' cases were randomly divided into the comparison/research group according to the surgery method. The two groups of patients were operated by the same medical team, and they were placed in a 90-degree lying position on the unaffected side, with a pillow under the armpit to increase the width of the intercostal space. The anesthesia method was general anesthesia with double-lumen tracheal intubation. During the operation, the affected lung was kept collapsed, and the contralateral lung was ventilated with one lung. Among them, the research group usually chose the fourth or fifth intercostal space of the anterior axillary line, which was determined according to the interlobar fissure, the hilum of the lung, and the location of the lesion. In comparison group, an incision of about 1.5 cm in length was made at the 7th or 8th intercostal space of the midaxillary line, and the trocar was placed as the observation hole, and the 3rd or 4th intercostal space between the anterior axillary line and the midaxillary line was selected as the main operation hole. The size of the incision was 3-4 cm, a soft incision protective sleeve was placed in the incision, and an incision of about 1.5 cm in length between the 7th or 8th intercostal space of the posterior axillary line was selected as the auxiliary operation hole. Both groups underwent segmentectomy and hilar and mediastinal lymph node dissection.

### 2.4. Outcome Measures

1. Perioperative indexes of the two groups (observation of intraoperative blood loss, operation time, and number of lymph node dissection). (2) Determination of tumor markers: after treatment, 5 ml of fasting elbow vein blood was drawn from the patient, the supernatant was centrifuged, and CYFRA21-1, CA125, as well as VGEF levels were measured by radioimmunoassay. (3) Immune function: after centrifugation of the above patients' serum, CD^4+^, CD^3+^, and CD^4+^/CD^8+^ were measured via flow cytometry (American BD company, FACS Vantage type). (4) Adverse reaction determination: record the occurrence of complications of the two groups of patients during treatment

### 2.5. Statistical Analysis

All data were discussed using SPSS 28.0 The measurement data were expressed via *x* ± *s*, and the intergroup data were tested by independent *t* test; *χ*^2^ test was adopted for counting data. *P* < 0.05, significant difference.

## 3. Results

### 3.1. General Data Comparison

The gender, average age, tumor diameter, pathological type, and other general data of the two groups of patients were compared by *t* test and chi-squared test, and there was no significant difference (*P* > 0.05). See Table 1.

### 3.2. Perioperative Improvement

There was no statistical difference between the two groups in terms of operative time and the number of lymph node dissection groups (*P* > 0.05). Patients in research group had lower surgical bleeding than comparison group, and this difference was statistically significant (*P* < 0.05). See Figure 1.

### 3.3. Comparison of Tumor Marker Levels

There was no significant difference in the levels of tumor markers between the two groups before treatment. After treatment, the levels of CYFRA21-1, CA125, and VGEF in the research group were significantly lower than comparison group, and the difference was significant (*P* < 0.05). See Figure 2.

### 3.4. Immune Level Comparison

There was no significant diversity in the immune level between the two groups before treatment (*P* > 0.05), while the differences in CD^4+^, CD^3+^, and CD^4+^/CD^8+^ after treatment were significant, and the research group was higher than comparison group (*P* < 0.05). See Figure 3.

### 3.5. Prognostic Complications

There was 1 case of postoperative pleural effusion and 1 case of postoperative air leakage in the study group, and 1 case of postoperative pulmonary infection in the control group. There was no statistical diversity in postoperative complications between the two groups (*P* > 0.05).

## 4. Discussion

NSCLC has become one of the most serious malignant tumors threatening human health in China. In addition, the physiological function of most patients declines, and the organs and tissues of various systems are aging, so the requirements for surgery are higher [11, 12]. The surgical treatment principle of NSCLC was to completely remove the tumor as far as possible and retain the healthy lung tissue as far as possible and perform corresponding lobectomy and systematic hilar and mediastinal lymph node dissection. Studies have found that for early-stage lung cancer with a diameter of less than 2 cm, segmentectomy had a similar long-term effect as lobectomy and preserves the patient's lung function to the greatest extent, while reducing related complications after lung resection [13]. Clinically, three-hole thoracoscopic lobectomy could remove the focus and gave play to the therapeutic effect [14]. In recent years, the technology of single-port thoracoscopic lobectomy had gradually matured, and many explorations have also confirmed the feasibility of single-port thoracoscopic segmentectomy [15]. In terms of operation time, postoperative extubation time, and complication rate, single-port thoracoscopic surgery is safe and reliable [16]. In addition, due to the incision was in an intercostal space, postoperative pain, chest wall paresthesia, and other discomforts were significantly reduced compared with traditional surgery [17]. On the premise that minimally invasive surgery was safe and feasible, the minimally invasive advantages of single-port thoracoscopy were more prominent, and the related lung function was protected [18]. The clinical application advantage of single-hole thoracoscopic lobectomy had become the focus of minimally invasive thoracic surgery [19].

The results of this study indicated that there was no remarkable diversity between the two groups in terms of operation time and the number of lymph nodes dissected during the operation. The surgical blood loss in research group was lower than in comparison group. The results indicated that single-hole thoracoscopic lobectomy had certain advantages in terms of surgical blood loss, which implied that single-hole thoracoscopic lobectomy, on the one hand, could select an operation hole between fourth, or fifth ribs according to the upper, middle, and lower lobe lesions, which could effectively reduce the number of incisions, reduce body trauma, reduce drainage flow, and shorten drainage time. On the other hand, when thoracoscopic accesses to the body, it was not easy to damage blood vessels, which could reduce bleeding [20].

Clinical imaging indicators are commonly used to evaluate the prognosis of patients, but imaging examination will be affected by the surrounding tissue, boundary, and volume of the lesion, and the requirements for imaging physicians and equipment are relatively high [21]. In addition, even if there is no progress in imaging results, the level of tumor markers may continue to rise [22]. Tumor markers usually exist in the blood, and their levels in host cells will also show certain changes. Because of the advantages of fast and simple detection, it has a good indication for the patient's condition development and efficacy evaluation [23]. VEGF is affirmed to participate in NSCLC angiogenesis and metastasis [24]. CYFRA21-1 is a soluble fragment of cytokeratin, which could be released into the blood, which has a high diagnostic value for patients with NSCLC [25]. Its detection level can be used to reflect the short-term efficacy of tumor treatment [26]. The results of this study exhibited that the improvement of the above tumor markers in the patients in the research group was less than comparison group, suggesting that the single-port thoracoscopic segmentectomy might reduce the generation of tumor markers and improve the prognosis of NSCLC.

T lymphocytes have the function of immune regulation and can produce a better stable effect on the immune internal environment of the body [27]. Among them, CD^8+^ can effectively reflect inhibitory T cells, CD^3+^ is a marker of mature T cells, and CD^4+^ can represent helper T cells. Compared with normal people, the level of T cell differentiation antigens such as CD^3+^, CD^4+^, and CD^4+^/CD^8+^ in cancer population is significantly lower [28]. Thus, the above indicators could effectively evaluate the level of autoimmunity [29]. The results of this study exhibited that the improvement of CD^3+^, CD^4+^, and CD^4+^/CD^8+^ in the research group after treatment was better than comparison group. This might be because single-port thoracoscopic segmentectomy could activate the immune response of the body, promote cell apoptosis, and to some extent, promote the killing function of new lymphocytes, so it could enhance the body immunity and improve the prognosis [30]. Furthermore, the outcomes discovered that the incidence of postoperative complications in research and comparison group was roughly similar, and there was no prominent diversity, indicating that single-port thoracoscopic segmentectomy possessed high safety and excellent clinical effect in the early treatment of NSCLC. In addition, this study should further explore the lung function, overall survival rate, and progression free survival rate of NSCLC patients via a single-port thoracoscopic segmentectomy to estimate the prognosis.

To sum up, single-hole thoracoscopic segmental resection could decrease intraoperative bleeding, reduce the level of serum tumor markers, and ameliorate immune function. Its clinical effect was superior to three-hole thoracoscopic segmental resection, which possessed certain clinical application value.

## Figures and Tables

**Figure 1:** Comparison of operation time, intraoperative blood loss, and number of lymph node dissection groups. (a) Operation time; (b) Intraoperative blood loss. (c) Number of lymph node dissection groups. ^##^*P* < 0.01 vs. comparison group.

**Figure 2:** Comparison of tumor marker levels between two groups of patients. (a) CYFRA21-1; (b) CA125; (c) VGEF. ^∗∗^*P* < 0.01 vs. before treatment, ^#/##^*P* < 0.05/0.01 vs. after comparison group.

**Figure 3:** Comparison of immune levels. (a) CD^4+^; (b) CD^3+^; (c) CD^4+^/CD^8+^. ^∗^*P* < 0.05 vs. before treatment, ^#^*P* < 0.05 vs. after comparison group.

**Table 1:** Comparison of general data between the two groups [*n*, ($\bar{x}\pm s$)].

Group	Gender (men/women)	Average age (age)	Tumor diameter (cm)	Pathological type	
				Adenocarcinoma	Squamous cell carcinoma
Comparison group (40)	28/12	56.87 ± 6.39	1.88 ± 0.23	33	7
Research group (40)	29/11	56.69 ± 6.23	1.89 ± 0.28	32	8
*χ* ^2^ */t*	0.061	0.023	0.074	0.065	0.346
*P*	0.805	0.731	0.941	0.799	0.556

## Data Availability

No data were used to support this study.
